# Proton-Binding Motifs of Membrane-Bound Proteins: From Bacteriorhodopsin to Spike Protein S

**DOI:** 10.3389/fchem.2021.685761

**Published:** 2021-05-31

**Authors:** Ana-Nicoleta Bondar

**Affiliations:** Freie Universität Berlin, Department of Physics, Theoretical Molecular Biophysics Group, Berlin, Germany

**Keywords:** hydrogen-bonding, proton transfer, proton antenna, membrane transporter, spike protein S

## Abstract

Membrane-bound proteins that change protonation during function use specific protein groups to bind and transfer protons. Knowledge of the identity of the proton-binding groups is of paramount importance to decipher the reaction mechanism of the protein, and protonation states of prominent are studied extensively using experimental and computational approaches. Analyses of model transporters and receptors from different organisms, and with widely different biological functions, indicate common structure-sequence motifs at internal proton-binding sites. Proton-binding dynamic hydrogen-bond networks that are exposed to the bulk might provide alternative proton-binding sites and proton-binding pathways. In this perspective article I discuss protonation coupling and proton binding at internal and external carboxylate sites of proteins that use proton transfer for function. An inter-helical carboxylate-hydroxyl hydrogen-bond motif is present at functionally important sites of membrane proteins from archaea to the brain. External carboxylate-containing H-bond clusters are observed at putative proton-binding sites of protonation-coupled model proteins, raising the question of similar functionality in spike protein S.

## Introduction

Proton transfer reactions are fundamental to cells from all branches of life. Among proteins that use proton binding and proton transfer for biological function, one of the best studied is bacteriorhodopsin, a small light-driven proton pump of the halophile archaeon *Halobacterium salinarium*. The first three-dimensional structure of bacteriorhodopsin, solved in 1975 by Henderson and Unwin using cryo-Electron Microscopy (cryo-EM), identified the seven transmembrane helices of the protein at a resolution of 7Å (Henderson and Unwin, 1975). In recent years, structures of bacteriorhodopsin solved with time-resolved serial femtosecond crystallography provided an atomic-resolution movie of structural changes during the proton-transfer reaction cycle (Nango et al., 2016; Weinert et al., 2019). Knowledge derived from simple model systems such as bacteriorhodopsin and other microbial rhodopsins can inform and guide studies of significantly more complex proteins and protein complexes that use protonation change and proton transfer during their reaction cycles (Ernst et al., 2014; Govorunova et al., 2017; Bondar and Lemieux, 2019). An example are the ASIC-like ion channels thought to participate in a cellular pH-sensing mechanism of specialized neurons (Jalalvand et al., 2016; Jalalvand et al., 2018). During ischemia and traumatic brain injury, a drop in extracellular pH and release of glutamate associate with hyperactive N-methyl-D-aspartate (NMDA) receptors and neuronal cell death (Regan et al., 2019).

pH sensing by proteins is thought to involve the chemical reaction of protonation change of a relatively small number of the titratable groups, typically carboxylate and histidine sidechains (Damaghi et al., 2013; Schönichen et al., 2013). Histidine sidechains, with their nominal pKa of 6.54 ± 0.4, can titrate at physiological values of cytosolic pH (Schönichen et al., 2013). The pKa value of an amino acid residue may, however, depend strongly on the environment (Thurlkill et al., 2006a). For example, whereas the nominal pKa values for aspartic and glutamic acids in solution are, respectively, 3.67 ± 0.4 and 4.25 ± 0.5 (Thurlkill et al., 2006b), pKa values as low as 1.56 ± 0.14 and as high as seven were determined with Nuclear Magnetic Resonance (NMR) for aspartic groups of the soluble protein PsbO (Gerland et al., 2020). In this perspective article, common proton-binding and H-bonding motifs are discussed with examples from simple model systems to more complex proteins.

### An Inter-helical Carboxylate-Hydroxyl H-Bond Motif Common to Membrane Transporters and Receptors

Membrane insertion of Asp/Glu groups is energetically costly, with apparent free energy penalties of ∼4–5 kcal/mol (Xie et al., 2007), and indeed there is only a relatively small probability that Asp and Glu locate in the hydrophobic core of *α*-helical membrane proteins (Ulmschneider and Sansom, 2001). Presence of carboxylates in transmembrane regions of membrane transporters and receptors is thus of direct interest to evaluate structure-function relationships, particularly for proteins in which these carboxylate groups could be involved in proton binding and proton transfer. Examples discussed here suggest that internal carboxylates used by membrane proteins for proton binding might be part of common inter-helical H-bond motifs; this could guide studies of other, more complex proteins for which proton-binding groups are yet to be identified.

A prominent example of a membrane transporter that uses internal carboxylates to bind protons is *bacteriorhodopsin*, which for decades has served as model system to study proton pumps (Lanyi, 1999; Herzfeld and Tongue, 2000; Balashov and Ebrey, 2001; Kandori, 2004; Kouyama et al., 2004; Gerwert et al., 2014). The primary proton acceptor group of bacteriorhodopsin is D85 (Metz et al., 1992), a carboxylate within one helical turn of T89, whose sidechain can serve as intermediate carrier for the proton transferred from the Schiff base proton donor to D85 (Bondar et al., 2004; Nango et al., 2016; Ni et al., 2018) (Figure 1A). Adjacent to T89, T90 has an inter-helical H-bond with D115, a carboxylate that stays protonated throughout the entire reaction cycle (Metz et al., 1992), and an intra-helical H-bond to the backbone carbonyl of W86 (del Val et al., 2014a). In the structure of the resting state of bacteriorhodopsin (Luecke et al., 1999), the cytoplasmic proton donor D96 (Gerwert et al., 1989) is within inter-helical H-bond distance from the T46 hydroxyl, which is within H-bond distance from the backbone carbonyl of F42 (Figure 1A); later during the reaction cycle, rearrangements of hydrophobic sidechains associate with formation of a water chain from D96 to the retinal Schiff base (Weinert et al., 2019). That is, at two internal sites where protons bind, bacteriorhodopsin can have inter-helical carboxylate-hydroxyl H-bonding and intra-helical H-bonding of the Thr hydroxyl group to a backbone carbonyl group (del Val et al., 2014a). The fact that only D96 changes protonation, whereas D115 remains protonated, suggests local protein environment other than with the direct H-bond partner impacts protonation change (del Val et al., 2014a). At the extracellular proton-release side, H-bonding between S193 and E204 depends on the protonation state (Gerwert et al., 2014).

**FIGURE 1:** Illustration of inter-helical carboxylate-hydroxyl H-bond motifs. For clarity, only selected backbone groups are shown. Numbers in blue represent H-bond distances in Å. **(A)** The bacteriorhodopsin proton pump, PDB ID:5ZIM (Hasegawa et al., 2018). **(B)** The viral ion channel OLPVR1, PDB ID:7AKY (Zabelskii et al., 2021). **(C)** EAAT1 bound to L-Asp substrate, PDB ID:5LLU (Canul-Tec et al., 2017). **(D)** The glutamate transporter VGLUT2, PDB ID:64VD (Li et al., 2020). **(E)** The LacY symporter, PDB ID:2V8N. **(F)** The HV1 proton channel, PDB ID:5OKK, molecule #7 (Bayrhuber et al., 2019). All molecular graphics were prepared with Visual Molecular Dynamics, VMD (Humphrey et al., 1996).

Similar inter-helical carboxylate-hydroxyl motifs were identified in structures of other membrane transporters, such as *the C1C2 channelrhodopsin chimera* and *the sodium pump rhodopsin KR2* (del Val et al., 2014b; Bondar and Smith, 2017; Siemers et al., 2019), the *SERCA calcium pump ATPase*, and *the multidrug transporter AcrB* (del Val et al., 2014a; Bondar and Lemieux, 2019), and can be observed in the recently solved structure of *viral rhodopsin OLPVR1*, a sodium/potassium ion channel (Zabelskii et al., 2021) (Figure 1B). Likewise, recently solved structures of *glutamate transporters VGLUT2* (Li et al., 2020) and *EAAT1* (Canul-Tec et al., 2017), which are members of families of neurotransmitter transporters essential for the functioning of the brain (Münster-Wandowski et al., 2016; Martineau et al., 2017), indicate inter-helical carboxylate-hydroxyl motifs at functionally important sites of both transporters: In the structure of VGLUT2, the putative pH sensor E191 (Li et al., 2020) H-bonds to S84 and T194 (Figure 1D); in EAAT1, D380 is within H-bond distance from T130 and thus close to M128, a group whose mutation to Arg inhibits glutamate transport (Chivukala et al., 2020); D456 H-bonds to the L-Asp substrate and to S343—which was noted as a conserved group whose mutation in wild-type EAAT1 inhibits transport (Canul-Tec et al., 2017); L-Asp H-bonds to three Ser/Thr hydroxyl groups (Figure 1C).

G-Protein Coupled Receptors (*GPCRs*) are membrane proteins that mediate communication between cells and their external environments. Protonation change might occur at carboxylate D2.50 (Zhang et al., 2015; Vickery et al., 2018), a carboxylate group part of the sodium-binding site in many class-A GPCRs (Katritch et al., 2014). H-bond networks conserved among static structures of GPCRs show D2.50 paired with S7.46, that is, a carboxylate-hydroxyl pair is present at a functionally important site (Bertalan et al., 2020) [the Ballesteros and Weinstein numbering scheme is used for GPCR groups (Ballesteros and Weinstein, 1995)].

Inter-helical H-bonding between Asp/Glu and Ser/Thr could provide an efficient mechanism to couple protonation change with local protein dynamics (Bondar and Smith 2017). Hydrophobic contacts of non-polar segments of these H-bond partners can reduce H-bond dynamics and strengthen H-bonding (Nemethy et al., 1963; Fernandez and Scheraga, 2003), and alteration of the pKa of an internal carboxylate might require local protein conformational change enabling water access to the carboxylate (Szaraz et al., 1994). In bacteriorhodopsin, the T90-D115 H-bond (Figure 1A) is in a local environment with more non-polar contacts than T46-D96, and its H-bond distance experiences smaller-amplitude fluctuations at room temperature (del Val et al., 2014a); the lesser hydrophobic packing near T46-D96 associates with water molecules entering rapidly the vicinity of D96 when the protein is mutated elsewhere (del Val et al., 2014a), and during the reaction cycle of the wild-type pump a file of waters assembles to bridge D96 to the Schiff base proton acceptor (Freier et al., 2011; Weinert et al., 2019).

Protonation change at an inter-helical carboxylate-hydroxyl pair might couple to altered local dynamics of the helix hosting the hydroxyl group: Ser/Thr hydroxyl groups can compete with backbone amide groups for H-bonding to a carbonyl group (Gray and Matthews, 1984; Presta and Rose, 1988), which increases local fluctuations of the helix (del Val et al., 2012). Alternatively, altered helix dynamics might impact local dynamics and hydration of the hydroxyl-carboxylate H-bond (Figure 2A).

**FIGURE 2:** Cartoon representation of inter-helical carboxylate-hydroxyl H-bonds and H-bond clusters. **(A)** The inter-helical carboxylate-hydroxyl H-bond may couple protonation change with changes in local protein dynamics (Bondar and Smith, 2017). **(B)** An internal carboxylate group and an external proton antenna cluster communicate via a water wire. **(C)** An interface H-bond cluster, as observed for spike protein S bound to ACE2 (Karathanou et al., 2020).

### Other H-Bond Motifs at Internal Proton-Binding Sites of Membrane Transporters

Local H-bonding and hydrophobic packing are likely key mechanisms used by proteins to control protonation of a proton-binding group–and different solutions as to which sidechain serves as H-bond partner for proton-transfer sidechains of membrane transporters appear to exist.

In *the plasma membrane proton pump AHA2*, which is a P-type ATPase, the primary proton donor/acceptor D684 (Buch-Pedersen and Palmgren, 2003) makes an inter-helical H-bond with an Asn (Pedersen et al., 2007; Guerra and Bondar, 2015; Focht et al., 2017); Likewise, OLPRV1, EAAT1, VGLUT2, and LacY, have at functionally important sites inter-helical bonds between Ser/Thr and Asn instead of Asp (Figure 1B–E).

In bacteriorhodopsin D212, which might functions as an intermediate proton carrier (Dioumaev et al., 1999; Phatak et al., 2009) has inter-helical H-bonds with Y57 and Y185 (Figure 1A), both important for optimal control of H-bond dynamics in the wild-type pump: mutating either Tyr group alters the kinetics of the reaction cycle (Rath et al., 1993; Govindjee et al., 1995), and Y57F has weak Y185-D212 H-bonding (del Val et al., 2014a). In the *Escherichia coli* proton-galactopyranoside symporter *LacY* E325, which deprotonates during the reaction cycle (Sahin-Toh and Kaback, 2001; Guan and Kaback, 2006), is part of a local H-bond network with Tyr and His sidechains (Figure 1E). Deprotonation of E325 causes protein structure changes that depend on the composition of the surrounding lipid bilayer (Andersson et al., 2012).

*Hv1*, also known as *HVCN1* (human voltage-gated proton channel) is a proton-selective ion channel whose action early after ischemia contributes to brain damage by providing the cancer cell with protons to compensate for the electron-transfer action of phagocytic cell NADPH oxidase (Wu et al., 2012). Proton selectivity of Hv1 requires a carboxylate group at D112 (Figure 1F), as some mutants with a neutral group instead Asp or Glu at this position loose proton specificity and became anion selective, and proton specificity could not be recovered when mutating D112 to His (Musset et al., 2011). That Hv1 becomes predominantly anion selective when its proton sensor is neutralized by mutation (Musset et al., 2011) resembles the behavior of bacteriorhodopsin, which from an outward proton pump becomes an inward chloride pump when the primary proton acceptor D85 is mutated to Thr (Sasaki et al., 1995), and underlines the need to decipher the role of electrostatic interactions–of static protein groups and of mobile ions, that govern charge states along the reaction cycle of ion transporters (Song and Gunner, 2014). The recent solution NMR structure of Hv1 reports for the sidechains of D112, R208, and R211 (Figure 1F) coordinates modeled by considering steric packing (Bayrhuber et al., 2019), and interactions of internal arginine sidechains can change in the presence of membrane voltage (Geragotelis et al., 2020). This suggests Hv1 has a rather dynamical internal H-bond network.

### H-Bond Networks of Histidine Sidechains at Proton-Binding Sites of Membrane Transporters and Receptors

Internal histidine groups can be central to the reaction mechanisms of protonation-coupled transporters and receptors. Examples include 1) H322 of LacY is part of an inter-helical H-bond motif with E325 at a proton-binding site (Figure 1D); 2) H128 of VGLU2 is thought to pick up a proton at the lumen side of the membrane, and connect to the E119 proton sensor via a water-filled pore (Li et al., 2020) (Figure 1); 3) H140 of Hv1 is a putative binding site for Zn^2+^ (DeCoursey et al., 2016; Bayrhuber et al., 2019), and its inter-helical H-bond partner D185 might be involved in ΔpH-gating (DeCoursey, 2018); 4) A pair of two H37 groups of the influenza channel M2 could participate in a proton-conductance mechanism that involves low-barrier H-bonding (Fu et al., 2020); 5) A cluster of histidine sidechains was proposed to ensure proton-sensing by the ovarian cancer GPCR 1, known as OGR1 or GPR68 (Ludwig et al., 2003; Holzer, 2009). OGR1, and other members of the proton-sensing GPCR subgroup, are activated when the extracellular pH becomes acidic, and histidine protonation couples with protein conformational change (Radu et al., 2004; Wang et al., 2004).

Taken together, the examples above suggest that internal histidine sidechains implicated in proton binding tend to be part of local H-bond clusters with carboxylate and/or other histidine sidechains. An Asp-His pair is also involved in pH sensing by the soluble protein hemoglobin (Srivastava et al., 2007).

### Carboxylate Clusters as Proton Antennas on Protein Surfaces

Proton antennas consist of clusters of closely spaced carboxylate, or of carboxylate and histidine groups, which can capture protons and prolong the time protons spend bound at the surface of the protein (Gutman and Nachliel, 1990; Sacks et al., 1998; Ädelroth and Brzezinski, 2004), and deliver a proton to a proton-entry site (Checover et al., 2001) (Figure 2B). Putative proton antenna clusters have been identified for bacteriorhodopsin (Checover et al., 2001), cytochrome *c* oxidase (Ädelroth and Brzezinski, 2004), and for the PsbO subunit of photosystem II (Shutova et al., 2007; Lorch et al., 2015; Kemmler et al., 2019). Surface carboxylates could be part of a pH-dependent conformational switch of PsbO (Bommer et al., 2016), and of a local buffering mechanism used by photosystem II to respond to acidification of the lumen (Gerland et al., 2020). The two carboxylate groups thought to bind the proton are part of a dynamic protein-water H-bond network that extends across the interface between PsbO and another protein subunit of photosystem II (Kemmler et al., 2019).

### H-Bond Networks of SARS-CoV-2 Protein S

The acidic environment of the endosome activates membrane fusion of coronaviruses, but it remains unclear whether acidity is required for proteases that cleave protein S to activate fusion, or for the spike protein itself (Heald-Sargent and Gallagher, 2012; Li, 2016). Membrane fusion might also be assisted by calcium binding to conserved negatively charged groups of SARS-CoV spike protein S (Millet and Whittaker, 2018).

Sequences of corona spike proteins S tend to carry significant net negative charges and contain patches rich in carboxylate, or carboxylate and histidine groups (Karathanou et al., 2020), but a discussion of a putative involvement of these patches in ion binding would be speculative. From graph-based analyses we discovered that titratable groups can participate in H-bond clusters that tend to have three-fold compositional symmetry when SARS-CoV-2 protein S is closed (Karathanou et al., 2020). Loss of this three-fold symmetry in the pre-fusion conformation could contribute to conformational selection of one protein S protomer to bind to the ACE2 receptor (Karathanou et al., 2020). An H-bond network that extends across the interface between the Receptor Binding Domain (RBD) of protein S and ACE2 contains N501 (Karathanou et al., 2020), which is mutated to Tyr in the United Kingdom virus variant (Leung et al., 2021). E484, which is mutated to Lys in the South African variant (Tegally et al., 2021), is close in sequence to RBD-Y449, which H-bonds to ACE2-D38 (Karathanou et al., 2020).

Elsewhere on the surface of protein S, intra-molecular H-bonding of D614 would be lost in the D614G virus variant (Korber et al., 2020); this mutation favors enhanced conformational dynamics of the spike protein, which could enable ACE2 binding (Benton et al., 2021). At the C-terminal region of the ectodomain of the closed protein S, a symmetrical H-bond cluster of no fewer than 33 protein groups includes six carboxylates and six histidine sidechains (Karathanou et al., 2020). Close to the R815 proteolytic cleavage site, E819 H-bonds to three Ser/Thr groups in all protomers of the closed and open conformations, and contributes to a large H-bond cluster in a pre-fusion protomer (Karathanou et al., 2020). Cryo-EM data suggest D830 and D843 are part of a pH-dependent switch that enables protein S to adopt, at low pH, a conformation incompatible with binding of particular antibodies (Zhou et al., 2020). Future experiments and computation are needed to evaluate any pH-dependent conformational changes at the interface between protein S and ACE2 (Figure 2C).

## Conclusion

Proteins across all branches of life rely on proton binding and proton transfer to exert their biological function. As three-dimensional structures of proteins and macro-molecular protein complexes involved in human physiology and disease become available, reasonable predictions of likely proton-binding sites and proton-transfer events are of interest to understand reaction mechanisms and potentially guide drug design. Simpler model proteins inform on H-bonding motifs common at proton-binding sites, and on structural elements that can shape the energetics of proton transfers in heterogeneous protein environments. Examples discussed here (Figure 1) illustrate an inter-helical H-bond carboxylate-hydroxyl motif that can ensure coupling between carboxylate protonation, protein conformational dynamics, and local water accessibility (Figure 2A). On the surface of the protein, carboxylate clusters may transiently bind a proton to then deliver it to an internal proton-binding site (Figure 2B) or for buffering, and participate in pH-dependent conformational switching that could impact protein interactions (Figure 2C). Dissecting the functional role of surface proton-binding clusters would need to account for local water interactions and protein conformational dynamics.

## Data Availability

Publicly available datasets were analyzed in this study. This data can be found here: Protein Data Bank, with accession codes as indicated in the article.
